# A Semantic Analysis and Community Detection-Based Artificial Intelligence Model for Core Herb Discovery from the Literature: Taking Chronic Glomerulonephritis Treatment as a Case Study

**DOI:** 10.1155/2020/1862168

**Published:** 2020-09-01

**Authors:** Yun Zhang, Yongguo Liu, Jiajing Zhu, Shuangqing Zhai, Rongjiang Jin, Chuanbiao Wen

**Affiliations:** ^1^Knowledge and Data Engineering Laboratory of Chinese Medicine, School of Information and Software Engineering, University of Electronic Science and Technology of China, Chengdu 610054, China; ^2^School of Basic Medical Science, Beijing University of Chinese Medicine, Beijing 100029, China; ^3^College of Health Preservation and Rehabilitation, Chengdu University of Traditional Chinese Medicine, Chengdu 610075, China; ^4^College of Medical Information Engineering, Chengdu University of Traditional Chinese Medicine, Chengdu 611137, China

## Abstract

The Traditional Chinese Medicine (TCM) formula is the main treatment method of TCM. A formula often contains multiple herbs where core herbs play a critical therapeutic effect for treating diseases. It is of great significance to find out the core herbs in formulae for providing evidences and references for the clinical application of Chinese herbs and formulae. In this paper, we propose a core herb discovery model CHDSC based on semantic analysis and community detection to discover the core herbs for treating a certain disease from large-scale literature, which includes three stages: corpus construction, herb network establishment, and core herb discovery. In CHDSC, two artificial intelligence modules are used, where the Chinese word embedding algorithm ESSP2VEC is designed to analyse the semantics of herbs in Chinese literature based on the stroke, structure, and pinyin features of Chinese characters, and the label propagation-based algorithm LILPA is adopted to detect herb communities and core herbs in the herbal semantic network constructed from large-scale literature. To validate the proposed model, we choose chronic glomerulonephritis (CGN) as an example, search 1126 articles about how to treat CGN in TCM from the China National Knowledge Infrastructure (CNKI), and apply CHDSC to analyse the collected literature. Experimental results reveal that CHDSC discovers three major herb communities and eighteen core herbs for treating different CGN syndromes with high accuracy. The community size, degree, and closeness centrality distributions of the herb network are analysed to mine the laws of core herbs. As a result, we can observe that core herbs mainly exist in the communities with more than 25 herbs. The degree and closeness centrality of core herb nodes concentrate on the range of [15, 40] and [0.25, 0.45], respectively. Thus, semantic analysis and community detection are helpful for mining effective core herbs for treating a certain disease from large-scale literature.

## 1. Introduction

Artificial intelligence is the general term of the modern technology of computer science [1], including image recognition [2], network analysis [3], and natural language processing [4]. Artificial intelligence technologies have been utilized in various fields of medicine, for example, automatic disease diagnosis [5], pathogenic network analysis [6], and biological text analysis [7] [8]. Meanwhile, Traditional Chinese Medicine (TCM) plays an important role and provides a unique theoretical and practical way to treat diseases for thousands of years in Chinese history. TCM has many treatments, such as acupuncture, medicinal wine, medicinal formula, and medicinal diet [9, 10]. Among them, medicinal formula, also called as the TCM formula, is the frequently used mode and is made up of several Chinese herbs. The TCM formula has many characteristics, such as compatibility combination, efficacy, treatment mechanism, and medication taboo [9, 11]. Compatibility combination can reflect the rationality of herb combination in formulae and guide TCM doctors to make up formulae [12], which mainly contains the “Sovereign-Minister-Assistant-Courier” combination rule and herb pair combination rule [13] [14]. Among them, the “Sovereign-Minister-Assistant-Courier” combination rule, also known as the “Jun-Chen-Zuo-Shi” combination rule, is a major combination principle of TCM formulae [15]. According to this principle, the sovereign herb plays a major role for dealing with main symptoms and syndromes of diseases, the minister herb helps the sovereign herb to strengthen herbal efficacy, and the assistant and courier herbs provide supporting function to reconcile formulae (e.g., reducing side effects) [15, 16]. Thus, the herbs acting as the sovereign or minister play a key role in terms of treating diseases, while others play an assistant role [16, 17]. In this way, the herbs serving as the sovereign or minister are viewed as core herbs in TCM formulae [17–19]. In other words, a formula contains multiple herbs, and core herbs play a critical therapeutic effect for treating diseases. Many formulae are collected in books, medical records, and scientific literature; however, most of them do not record their core herbs [19], which is difficult for young doctors and learners to master the core concern of formulae and prescribe effective formulae for treating different diseases. Thus, discovering core herbs can help doctors and learners to understand the quintessence of formulae quickly and provide evidences and references for the clinical application of herbs and formulae [16, 18, 19]. Through discovered core herbs, doctors can optimize the herb combination of formulae and synergize herb efficacies to prescribe more effective formulae for treating diseases [15], [19].

In general, researchers mainly explored core herbs by manual analysis [20–22], data analysis [19, 23–27], and clinical and pharmacology experiments [16, 28]. The traditional way to discover core herbs is the manual analysis on TCM books. Researchers first collected the relative books about the TCM treatment of a certain disease and then explored the possible relations between herbs and this disease. Finally, they discovered core herbs according to frequent relations, which is suitable for small-scale researches [20–22]. Recently, researchers utilized data analysis methods, such as statistical approach, association rule, mutual information, and entropy clustering, to analyse the frequency of herbs and their cooccurrence relations in formulae for discovering herbal compatibility rules and core herbs from medical records [19, 23–27]. Data analysis approaches can deal with large-scale medical records; however, they need structured data. It is known that medical records contain personal information (e.g., name, age, and sex), diagnostic information (e.g., laboratory index, symptom, syndrome, and disease), and treatment information (e.g., western drug, Chinese herb, formula, and medical advice) [29] [30]. In order to discover core herbs for treating a certain disease, researchers must extract partial diagnostic and treatment information from large-scale records, which costs more time. Meanwhile, it is worth noting that existing core herb discovery models cannot understand the inner meanings and functions of herbs in these records [19, 23–27]. For example, herb *liquorice root* (Gan Cao) has many attributes, such as usage, efficacy, and taboo; however, existing models only consider the characters of Chinese words as text, then they cannot capture the implicit characteristics of this herb. In clinical experiments, researchers evaluated the efficacy of different herb combinations of TCM formulae on subjects to find effective herbs as core herbs [28]. In pharmacology experiments, researchers designed evaluation indexes, such as the network recovery index, to measure the scores of different ingredients in TCM formulae to find high score ingredients and considered the herbs with these ingredients as core herbs [16]. The experimental ways focus on few classical formulae and can analyse herb components in clinical trial and microscopic analysis perspectives to achieve high accuracy. However, enumerating all potential herb combinations and ingredients in an experimental way maybe impossible.

Besides books and medical records, there is rich scientific literature containing medical knowledge about TCM formulae [31]. To our best knowledge, there are few researches about discovering core herbs from the scientific literature. We consider some reasons: (1) literature is unstructured text, where disease, formula, and herb information are unevenly distributed in full text and cannot be processed easily; (2) it is hard to analyse the semantics of herbs in the literature; and (3) there are no good ways to represent herb semantics. Minority researchers studied classical literature to mine treatment patterns [32, 33], but they also process them artificially to deal with problem (1). However, they also do not analyse the inner meanings and functions of herbs in the literature for problems (2) and (3). In order to mimic the human learning mode for relatively accurately comprehending the literature and improve the efficiency of literature analysis, we introduce semantic analysis and community detection to handle these problems for analysing large-scale literature and discover core herbs efficiently.

In this paper, we propose an artificial intelligence model CHDSC for discovering the core herb for treating a certain disease based on semantic analysis and community detection, whose framework is shown in Figure 1. CHDSC mainly contains two artificial intelligence modules, in which a semantic analysis module is a natural language processing algorithm for analysing the semantics of herbs in large-scale literature by a Chinese word embedding algorithm ESSP2VEC as described in Section 3.1, and the community detection module is a network analysis algorithm to discover herb communities in the herbal semantic network by a label propagation-based algorithm LILPA as described in Section 3.2. The herbal semantic network is constructed by the semantic similarity of herbs based on the results of the semantic analysis module. The semantics of herbs contain which disease can be treated and how is it treated, then the herbal semantic network can reflect the relations between herbs and disease. Herbs in each community have the same or similar efficacy for treating multiple syndromes of a certain disease. Further, we consider important herbs in each herb community as the core herbs for treating the syndromes characterized by the community.

In order to validate the proposed model, we choose chronic glomerulonephritis (CGN) and discover the core herbs for treating this disease as a case study. Chronic Kidney Disease (CKD) is a class of kidney diseases with proteinuria, oedema, and haematuria as clinical symptoms [34]. The overall prevalence of CKD is 10.8%, and the number of patients in China is up to about 119.5 million [34]. CGN is a typical disease of CKD, which has different symptoms, such as oedema, haematuria, anaemia, albuminuria, and kidney function decrease and may lead to different degrees of renal dysfunction and chronic renal failure. CGN may damage heart function and the central nervous system and threaten life when it is severe [35]. In TCM, CGN is mainly recognized as the syndrome of qi deficiency of the spleen and kidney, the syndrome of deficiency of both qi and yin, the syndrome of yin deficiency of the liver and kidney, the syndrome of yang deficiency of the spleen and kidney, and the syndrome of liver depression and qi stagnation [36]. In addition, CGN also contains the syndrome of fluid-dampness, the syndrome of dampness-heat, the syndrome of blood stasis, and the syndrome of damp-turbidity [36]. It is shown that TCM treatment can improve and recover renal function and alleviate clinical symptoms [37]. Thus, discovering core herbs in TCM formulae for CGN treatment is helpful for improving the curative effect and precisely prescribing medicine. TCM doctors can utilize effective core herbs to form new formulae for treating different syndromes of patients with CGN.

In order to discover core herbs for treating different syndromes of CGN, we propose CHDSC with three stages: corpus construction, herb network establishment, and core herb discovery. The literature of CGN treatment in TCM is acquired from the China National Knowledge Infrastructure (CNKI). In the first stage, the CGN corpus is constructed by preprocessing the collected large-scale literature. In the second stage, a semantic analysis module based on word embedding is proposed by integrating the stroke, structure, and pinyin features of Chinese characters to analyse the semantics of herbs in literature, then the semantic similarity among herbs is measured, and a herbal semantic network is built according to semantic similarity. In the last stage, a community detection module based on label propagation is used to discover herb communities and core herbs in the herbal semantic network. We also analyse the community size, degree, and closeness centrality distributions of the network to mine the rules of core herbs. Experimental results show that CHDSC uncovers three major herb communities where herbs in each community can be used for treating multiple syndromes of CGN, and discovers the core herbs for curing different syndromes of CGN with high accuracy. Core herbs mainly exist in the herb communities with more than 25 herbs. The degree and closeness centrality of core herb nodes in the herb network concentrate on the range of [15, 40] and [0.25, 0.45], respectively.

## 2. Related Work

In general, there are three type ways to discover core herbs: manual analysis, data analysis, and clinical and pharmacology experiments.

In manual analysis, researchers searched Chinese books about the TCM treatment of a specified disease, extracted corresponding formulae, and found core herbs by hand. Wang [20] investigated some classical books such as Shen-Nong-Ben-Cao-Jing and Huang-Di-Nei-Jing to discuss the methods for exploring the sovereign, minister, assistant, and courier herbs. Wang and Wang [21] analysed the compatibility and function of Zhi-Gan-Cao-Tang and found that *liquorice root* (Gan Cao) is its core herb with the efficacy of making up qi, blood, yin, and yang. Song and Niu [22] drew the rules on the determination of the sovereign herbs of Xie-Xin-Tang and analysed its sovereign herbs.

In data analysis, researchers discovered core herbs based on the frequency of herbs and their cooccurrence relations in datasets. Meanwhile, most studies focused on medical records. Zhou et al. [19] proposed an Effect Degree- (ED-) based algorithm to discover core herbs and compatibility rules with three steps: core herb discovery based on ED, network construction based on pointwise mutual information, and herb compatibility rule detection. They found 42 core herbs for treating consumptive lung disease. Zhan et al. [23] collected CGN treatment data in a Chinese biomedical literature database and mined the relationship among symptoms, syndromes, herbs, and formulae by the stratification algorithm based on keyword frequency, then they discovered that *milkvetch root* (Huang Qi), *danshen root* (Dan Shen), and *Indian bread* (Fu Ling) are core herbs. Ma et al. [24] extracted herbs, therapies, syndromes, and diseases in TCM formulae from medicine records and built a relation graph by NetDraw. The degree and closeness centrality were calculated to discover core herbs, then they found nine core herbs for treating gastric abscess. You et al. [25] established a formula database of bone marrow suppression treatment with a TCM kidney-tonifying method after radiotherapy and chemotherapy and applied cluster techniques and association rules to analyse medication rules. They found that *milkvetch root* (Huang Qi), *atractylodis macrocephalae rhizoma* (Bai Zhu), and *ligustri lucidi fructus* (Nv Zhen Zi) are frequently used herbs. Most data analysts also discovered the compatibility rules and treatment patterns of TCM formulae where core herbs are contained. Chen et al. [26] mined symptom-herb patterns with the triangular relationship of symptoms, syndromes, and herbs from medical records. They found the main symptom-herb patterns on four real-world patient records (insomnia, diabetes, infertility, and Tourette syndrome). Chang et al. [27] investigated the treatment patterns among stroke patients by a nationwide population-based study using random samples of one million individuals from the national health insurance research database in Taiwan. They found that Bu-Yang-Huan-Wu-Tang and *danshen root* (Dan Shen) are commonly used.

In clinical and pharmacology experiments, researchers analysed effective herb combinations or ingredients of a given formula to explore core herbs for treating a certain disease. Yan et al. [28] proposed a study protocol to explore the core herbs for treating primary insomnia in TCM, in which they performed a triple-blind, randomized, and parallel-group clinical trial to analyse the formulae of prestigious TCM clinicians and used association rules to find effective core herbs. Wu et al. [16] identified the roles of “Sovereign-Minister-Assistant-Courier” of herbs in the Qi-Shen-Yi-Qi formula for treating myocardial ischemia by the network pharmacology approach. They integrated disease-associated genes and protein-protein interaction experiments to construct an organism disturbed network of myocardial ischemia and developed a network-based index, Network Recovery Index (NRI), to measure the therapeutic efficacy of the Qi-Shen-Yi-Qi formula. As a result, the whole formula gets the NRI score of 864.48 and outperforms a single herb. Additionally, *danshen root* (Dan Shen) and *milkvetch root* (Huang Qi) obtain the NRI scores of 734.31 and 680.27, respectively; thus, the two herbs are regarded as core herbs.

The above researches obtain good results for discovering core herbs; however, manual analysis and medical experiments need high cost for large-scale samples. Meanwhile, for data analysis, researchers need to process medical records manually to obtain structured data. Data analysis methods are based on cooccurrence relations and do not contain the inner meaning of herbs in medical records. On the other hand, there is large-scale literature containing the domain knowledge of formulae. In this paper, we focus on analysing literature and introduce semantic analysis and community detection to analyse the meanings of herbs in the literature to discover core herbs for treating a disease in TCM.

## 3. Artificial Intelligence Module

In this section, we introduce the semantic analysis and community detection modules used in CHDSC for core herb discovery. Firstly, we propose a Chinese word embedding algorithm ESSP2VEC to deal with large-scale literature and analyse the semantics of herbs based on the stroke, structure, and pinyin features of Chinese characters by predicting the contextual words of Chinese words. Secondly, we adopt a label importance-based label propagation algorithm LILPA to detect herb communities and core herbs, in which labels are propagated according to label importance based on node importance and node attraction. If the nodes own the same label when LILPA ends, they are allocated to the same community.

### 3.1. Word Embedding Algorithm

In order to analyse the semantics of herbs in large-scale literature, we propose the Chinese word embedding algorithm ESSP2VEC. We consider that it is a suitable model for learning the meanings of herbs from large-scale literature to handle problems (1) and (2). Word embedding is utilized to analyse word meanings based on the distributional hypothesis that similar words tend to appear in similar contexts; in other words, the semantics of words are included in their contextual words [38, 39]. Words are expressed as semantic word vectors, then we can consider that the meanings of words are contained in them [39]. In order to understand semantic word vectors intuitively, we take an example to visual some words in a two-dimensional surface by their semantic word vectors. As shown in Figure 2, semantic word vectors can contain some meanings of words and better distinguish different types of words, such as the animals (pig, sheep, and cow), the plants (tree and grass), and the actions (swim and dive). Thus, word embedding can capture the semantics of words to a certain degree. In collected large-scale literature, we can analyse the semantics of herbs and express them as semantic word vectors, which is a way to improve problem (3) to embody the semantics of herbs.

Further, herbs in the collected literature are recorded as Chinese words. Chinese words are made up of Chinese characters, which contain many semantically related internal features [40] [41]. Researchers proposed many Chinese word embedding algorithms for analysing the meanings of Chinese words by exploiting the character feature of Chinese words [42] and the internal features of Chinese characters, such as radical [43], component [44], stroke *n*-grams [39], structure [40], and pinyin [40]. Here, we introduce these features briefly.

- *Character* (https://en.wikipedia.org/wiki/Chinese_characters): characters are logogram developed for the writing of Chinese, which makes up Chinese words [42].
- *Radical* (https://en.wikipedia.org/wiki/Radical_(Chinese_characters)): radical is the first stroke or morphological component of Chinese characters, which is the catalogue of symbols that are classified according to the structure and meaning of Chinese characters in a dictionary [43].
- *Component*: component is a character-forming unit and has the function of assembling Chinese characters [44].
- *Stroken-gram* (https://en.wikipedia.org/wiki/Stroke_(CJK_character)): stroke is the uninterrupted dots and lines of various shapes that compose Chinese characters, such as horizontal, vertical, left-falling, right-falling, and turning, which is the smallest constitutional unit of Chinese characters. Stroke *n*-gram is the combination of strokes according to stroke order (https://en.wikipedia.org/wiki/Stroke_order) [39].
- *Structure*: structure is the azimuth relationship (13 patterns) among strokes, such as left-right and left-middle-right [40].
- Pinyin (https://en.wikipedia.org/wiki/Pinyin): pinyin is the romanization of Chinese characters, which consists of initials, finals, and tones [40].

However, existing researches do not consider these features together. Stroke *n*-grams include radical and component features and can capture partial semantics of the entire character [39] [40]. Meanwhile, the structure feature can capture the implication meanings of characters, and the pinyin feature can help us to understand the meanings of onomatopoeia and distinguish the characters which have the same stroke *n*-gram and structure [40]. Then, we can catch relatively comprehensive semantics of Chinese characters from the stroke *n*-gram, structure, and pinyin features. Thus, we propose ESSP2VEC to integrate the stroke *n*-gram, structure, and pinyin features of Chinese characters for analysing the semantics of Chinese words.

The architecture of ESSP2VEC is shown in Figure 3 with an explanatory example. In this example, we have a sentence “carry forward the spirit of laborious struggle vigorously,” where the target word is “laborious (https://www.zdic.net/hans/%E8%89%B0%E8%8B%A6),” which is made up of two Chinese characters, and its contextual words are “vigorously,” “carry forward,” “struggle,” and “spirit.” ESSP2VEC consists of input, feature extraction, feature encoding, ensemble feature, and output layers.

- *Input layer*: input layer is used to receive the target word *w*_*t*_.
- *Feature extraction layer*: this layer is used to decompose word *w*_*t*_ to independent characters and extract the stroke, structure, and pinyin of each character.
- *Feature encoding layer*: this layer is used to encode the stroke, structure, and pinyin features. We adopt the code defined in [40] to encode the stroke, structure, and pinyin features.
- *Ensemble feature layer*: this layer is designed to generate stroke *n*-gram (all combinations of stroke) by moving a slide window with different lengths on the stroke sequence as shown in Figure 3 and integrate stroke *n*-gram, structure, and pinyin features.
- *Output layer*: output layer is designed as a *softmax* layer [45] to calculate the probability that the contextual words of word *w*_*t*_ are predicted based on the ensemble features of word *w*_*t*_.

Similar to [39–45], we predict the contextual words based on the target word in ESSP2VEC. In particular, the target word is expressed as its ensemble features. Given corpus *C* represented as the sequence of words *w*_1_, ⋯, *w*_*t*_, ⋯, *w*_*N*_word__ formally, where the word *w*_*t*_ is the target word and *N*_word_ is the number of words. The set of the contextual words of word *w*_*t*_ is represented as

(1) $$\begin{array}{c} C_{t}=\left\{w_{t+i}\right\},\left(i\in \left[-c,0\right)\cup \left(0,c\right]\right), \end{array}$$

where *c* is the size of the contextual words and word *w*_*c*_ represented the element of *C*_*t*_, *w*_*c*_ ∈ *C*_*t*_, then the objective of ESSP2VEC is to maximize the log-likelihood in equation (2) where we hope to get the maximization of possibility *p*(*w*_*c*_ | *w*_*t*_), that is, word *w*_*c*_ can be predicted correctly with maximum possibility based on the target word *w*_*t*_.

(2) $$\begin{array}{c} L=\frac{1}{N_{\text{word}}}\overset{N_{\text{word}}}{\underset{t=1}{\sum }}\underset{w_{c}\in C_{t}}{\sum }\log p\left(w_{c}\;|\;w_{t}\right). \end{array}$$

Then, the *softmax* function is used to model probability *p*(*w*_*c*_ | *w*_*t*_) of predicting word *w*_*c*_ given word *w*_*t*_, which is defined as

(3) $$\begin{array}{c} p\left(w_{c}\;|\;w_{t}\right)=\frac{e^{s\left(w_{t},w_{c}\right)}}{\sum_{j=1}^{N_{\text{word}}}e^{s\left(w_{t},w_{j}\right)}}, \end{array}$$

where *s*(*w*_*t*_, *w*_*c*_) is a scoring function to map the pairs of word *w*_*t*_ and word *w*_*c*_ to a real number.

Chinese characters with similar stroke *n*-gram, structure, and pinyin may have similar semantics [40]. Thus, Chinese characters having similar ensemble features should have similar senses. Then, we define *s*(*w*_*t*_, *w*_*c*_) as equation (4) to calculate their similarity based on the ensemble features of word *w*_*t*_ and its contextual word *w*_*c*_, where *F*(*w*_*t*_) denotes the collection of the stroke *n*-grams of word *w*_*t*_; *v*_stroke *n*‐gram_, *v*_structure_, and *v*_pinyin_ are the embeddings of stroke *n*-gram, structure, and pinyin features, respectively; and *v*_*w*_*c*__ is the initial semantic word vector of word *w*_*c*_. By replacing *w*_*c*_ as *w*_*j*_, we also can compute *s*(*w*_*t*_, *w*_*j*_).

(4) $$\begin{array}{c} s\left(w_{t},w_{c}\right)=\left(\left(\underset{\text{stroke }n‐\text{gram}\in F\left(w_{t}\right)}{\sum }v_{\text{stroke }n‐\text{gram}}\right)+v_{\text{structure}}+v_{\text{pinyin}}\right)∙v_{w_{c}}. \end{array}$$

We optimize the objective function of equation (2) based on standard gradient methods [39]. After the training process, the semantic word vectors of contextual words are the output. Thus, we can obtain semantic word vectors *U* = {*u*_1_, ⋯, *u*_*t*_, ⋯, *u*_*N*_*n*word__} of all words in the corpus, where *u*_*t*_ denotes the semantic word vector of word *w*_*t*_ and *N*_*n*word_ is the number of nonrepetitive words in the corpus. By training ESSP2VEC in the collected large-scale literature corpus, we can analyse the semantics of herbs and express them as semantic word vectors.

There also are word embedding algorithms designed for other languages. For example, Park et al. [46] proposed a Korean word embedding algorithm, which uses *jamo* feature of Korean characters to construct the *jamon*-gram of Korean words and predict the contextual words of the target word based on its *n*-gram. Korean characters can be decomposed into *jamos* in turn, which are the smallest lexicographic units representing the consonants and vowels [46]. The *jamo* feature is extracted to construct the *jamon*-gram of Korean words, which is similar to the stroke *n*-gram of Chinese words. Then, the model predicts the contextual words of the target word based on its *jamon*-gram to obtain final word embeddings. For English, Bojanowski et al. [47] proposed the FastText algorithm to capture the subword feature of English words to construct character *n*-gram and predict the contextual words of the target word based on its character *n*-gram. English words can be divided into 26 alphabets, which are the smallest component units of English words. Different character combinations can form different features, such as etyma, prefixes, and suffixes, which contain part semantics of words [47]. The subword feature is extracted to construct the character *n*-gram of English words, which is similar to the stroke *n*-gram of Chinese words. For example, the 3-grams of the word *where* are *<wh*, *whe*, *her*, *ere*, *re>* [47]. Then, FastText predicts the contextual words of the target word based on its *n*-gram to obtain final word embeddings.

The above three methods both generate the *n*-gram of one feature of the target word (i.e., the stroke *n*-gram of Chinese, the *jamon*-gram of Korean, and the character *n*-gram of English) and predict the contexts of the target word based on its *n*-grams. For the proposed algorithm, ESSP2VEC not only constructs the stroke *n*-gram of Chinese words but also integrates the other two features (structure and pinyin) to analyse relatively comprehensive semantics of Chinese words. That is, ESSP2VEC considers both the morphological and phonetic features of Chinese words. Meanwhile, ESSP2VEC considers the similarity between the contextual words and the internal features of the target word to conduct prediction.

### 3.2. Label Propagation-Based Algorithm

According to the theory of ESSP2VEC, we can analyse the semantics of herbs and obtain their semantic word vectors. However, how to use the semantic word vectors to find core herbs is a challenge. In order to discover core herbs for treating a certain disease by the semantic word vectors, we first compute the semantic similarity among herbs and construct a herbal semantic network, where herbs are considered as nodes and if the semantic similarity between two herbs is larger than the average value of all similarity among herbs (threshold value), edges are formed between the two herbs. Then, we adopt a label importance-based label propagation algorithm LILPA [48] to detect communities in the herbal semantic network, which can further improve problem (3). Herbs in a community may have the same or similar efficacy and can treat multiple syndromes of a certain disease. Finally, we identify important nodes in each community as core herbs for treating the syndromes of the disease. Here, we introduce LILPA briefly.

There are many real-world networks, such as social networks, collaboration networks, and herb networks, in which nodes represent objects and edges represent their relations [18]. Real-world networks often consist of subnetworks or communities with nodes more tightly linked with respect to the rest of the networks [3]. Community detection can be informally considered as a problem of finding such communities in networks, which aims at assigning community labels to nodes such that the nodes in the same community share higher similarity than the nodes in different communities [49] [50]. Communities in networks are the division of networks into the groups of nodes having dense intraconnections and sparse interconnections [51]. In other words, the connections among nodes in communities are dense, while the connections between communities are sparse. Thus, community detection focuses on discovering communities with dense connection nodes in networks. If the nodes own the same label when the algorithm ends, these nodes are allocated to the same community.  Table 1 shows the corresponding concepts between core herb discovery and LILPA.

An example is given in Figure 4 to explain the process of community detection based on label propagation. Node *v*_6_ is chosen to update its labels firstly. Its neighbour nodes *v*_3_, *v*_4_, *v*_5_, *v*_8_, *v*_10_ launch their own label with belonging coefficient to node *v*_6_ (we assume that the belonging coefficient equals to 1). Then, node *v*_6_ receives labels (purple, 1), (purple, 1), (purple, 1), (green, 1), and (orange, 1). By normalizing their belonging coefficients, we obtain node *v*_6_ with labels (purple, 0.6), (green, 0.2), and (orange, 0.2). If the belonging coefficient is smaller than 1/*R* (we assume the filtering threshold *R* = 2), then the green and orange labels are filtered. Finally, the label of node *v*_6_ is updated to the purple label, so node *v*_6_ is assigned to purple community. Then, other nodes are chosen to update their labels. The above process is conducted continuously until the labels of nodes are kept unchanged. Finally, community detection is finished, and we can discover three communities in the example network. That is, nodes *v*_1_, *v*_2_, *v*_3_, *v*_4_, *v*_5_, *v*_6_ are assigned to a community; nodes *v*_7_, *v*_8_, *v*_9_ are assigned to a community; and nodes *v*_10_, *v*_11_, *v*_12_, *v*_13_ are assigned to another community. We can find that intercommunal relations among communities are sparser than the connections within the communities. In each community, the nodes with a large degree (the number of neighbours) are considered as important nodes, such as *v*_3_, *v*_8_, and *v*_10_. In addition, nodes are drawn in a layout area.

Given an undirected and unweighted network *G* = (*V*, *E*), where *V* = {*v*_1_, ⋯, *v*_*i*_, ⋯, *v*_*N*_node__} represents the set of nodes and *E* = {*e*_1_, ⋯, *e*_*i*_, ⋯, *e*_*M*_edge__} represents the set of edges. *N*_node_ and *M*_edge_ are the number of nodes and edges, respectively. The neighbour nodes of node *v*_*i*_ are expressed as *Z*(*v*_*i*_) = {*v*_*j*_ | *e*_*v*_*i*_*v*_*j*__ ∈ *E*}, and its degree is expressed as *k*_*v*_*i*__. The labels of node *v*_*i*_ are stored in *B*(*v*_*i*_) = {(*l*_1_^*i*^, *c*_1_^*i*^), ⋯, (*l*_*j*_^*i*^, *c*_*j*_^*i*^), ⋯, (*l*_*H*_^*i*^, *c*_*H*_^*i*^)}, where label *l*_*j*_^*i*^ is the *j*th label with a belonging coefficient *c*_*j*_^*i*^ of node *v*_*i*_, ∑_*j*=1_^*H*^*c*_*j*_^*i*^ = 1, and *H* is the number of labels in *B*(*v*_*i*_). The community characterized by label *l* is expressed as *O*^*l*^. Nodes are drawn in a rectangle layout area with length *L* and width *W*. The position and displacement of node *v*_*i*_ in the layout are denoted as ${\vec{P}}_{v_{i}}$ and ${\vec{D}}_{v_{i}}$, respectively.

In the above example, node *v*_6_ is randomly chosen to update its labels. In order to fix the updating order of nodes to improve stability, node importance is defined to reflect the weight of nodes in networks as

(5) $$\begin{array}{c} I_{v_{i}}=C_{v_{i}}\times k_{v_{i}}+\underset{v_{j}\in Z\left(v_{i}\right)}{\sum }\frac{k_{v_{j}}}{\sum_{v_{k}\in Z\left(v_{i}\right)}k_{v_{k}}}\times C_{v_{j}}\times k_{v_{j}}, \end{array}$$

where *C*_*v*_*i*__ = (*N*_node_ − 1)/∑_*v*_*j*_∈*V*_*d*_*v*_*i*_*v*_*j*__ is the closeness centrality of node *v*_*i*_ to measure its centrality in networks and *d*_*v*_*i*_*v*_*j*__ is the shortest distance between nodes *v*_*i*_ and *v*_*j*_.

Communities are the clusters of nodes owning dense intraconnections and sparse external connections [49]. In order to increase the attraction among nodes to obtain dense internal connection, the node attraction between nodes *v*_*i*_ and *v*_*j*_ is defined as

(6) $$\begin{array}{c} F_{v_{i}v_{j}}^{A}=\frac{x_{v_{i}v_{j}}^{2}}{\sqrt{\left(W\times L\right)/N}}, \end{array}$$

where *x*_*v*_*i*_*v*_*j*__ is the straight-line distance between nodes *v*_*i*_ and *v*_*j*_ in the layout area calculated by the positions of nodes in the layout area, which is different with *d*_*v*_*i*_*v*_*j*__ which is the shortest distance between nodes *v*_*i*_ and *v*_*j*_ calculated by the edge weight of networks.

When label *l* with a belonging coefficient *c* is sent from node *v*_*j*_ to node *v*_*i*_, the weight of this label is influenced by the node importance of sender, propagation distance (related to the node attraction among nodes), and its belonging coefficient [18]. Then, label importance is defined to measure the weight of labels of a node when they reach other nodes as

(7) $$\begin{array}{c} {LP}_{l,v_{j}\to v_{i}}=I_{v_{i}}\times c\times \sqrt{F_{v_{i}v_{j}}^{A}}. \end{array}$$

The processes of LILPA consist of initialization, node choice, node movement, label launch, label acceptation, termination judgement, and postprocess, as shown in Figure 5.

**Step 1 .**

Initialization. Nodes are allotted with labels (e.g., node's id) and random positions, then the node importance of all nodes is computed.

1. Set $S=V,B\left(v_{i}\right)=\left\{\left(l_{1}^{i}=i,c_{1}^{i}=1\right)\right\},\vec{P_{v_{i}}}=\left(x_{i}\in \left[-\left(L/2\right),L/2\right],y_{i}\in \left[-\left(W/2\right),W/2\right]\right)$, and $\vec{D_{v_{i}}}=\vec{0}$ for *v*_*i*_ ∈ *V*, *r* = 1, and *t* = 1. Here, *S* represents the node set where nodes have not been updated
2. Node importance is calculated, then the nodes in *S* are ordered in ascending order of node importance.

**Step 2 .**

Node choice. Node *v*_*i*_ is chosen to update its labels, which satisfies *I*_*v*_*i*__ = min(*I*_*v*_*j*__ | *v*_*j*_ ∈ *S*), then set *B*(*v*_*i*_) = ∅. Nodes with small importance can be influenced by nodes with large importance easily [18], then the labels of nodes with small importance are preferentially updated.

**Step 3 .**

Node movement. Node *v*_*i*_ moves to a new position according to its displacement.

(1) The displacement of node *v*_*i*_ is calculated by
  (8) $$\begin{array}{c} {\vec{D}}_{v_{i}}=-\underset{v_{j}\in Z\left(v_{i}\right)}{\sum }\frac{{\vec{P}}_{v_{i}}-{\vec{P}}_{v_{j}}}{\left|{\vec{P}}_{v_{i}}-{\vec{P}}_{v_{j}}\right|}\times F_{v_{i}v_{j}}^{A}+\underset{v_{j}\in Z\left(v_{i}\right)}{\sum }\frac{{\vec{P}}_{v_{i}}-{\vec{P}}_{v_{j}}}{\left|{\vec{P}}_{v_{i}}-{\vec{P}}_{v_{j}}\right|}\times F_{v_{i}v_{j}}^{R},\\ F_{v_{i}v_{j}}^{R}=\frac{W\times L}{N\times x_{v_{i}v_{j}}} \end{array}$$
(2) The position of the node is updated by
  (9) $$\begin{array}{c} {\vec{P}}_{v_{i}}={\vec{P}}_{v_{i}}+\frac{{\vec{D}}_{v_{i}}}{\left|{\vec{D}}_{v_{i}}\right|}\times \min\left(\left|{\vec{D}}_{v_{i}}\right|,\frac{\min\left(W,L\right)}{4}\right) \end{array}$$
(3) If node *v*_*i*_ is out of the layout area, then its position is restricted in the layout area by equations (10) and (11)
  (10) $$\begin{array}{c} x_{v_{i}}=\min\left(\frac{L}{2},\max\left(-\frac{L}{2},x_{v_{i}}\right)\right), \end{array}$$
  (11) $$\begin{array}{c} y_{v_{i}}=\min\left(\frac{W}{2},\max\left(-\frac{W}{2},y_{v_{i}}\right)\right) \end{array}$$

**Step 4 .**

Label launch. In this step, every node in the neighbouring nodes of node *v*_*i*_ sends its label with the maximal belonging coefficient to node *v*_*i*_.

1. For node *v*_*j*_ in *Z*(*v*_*i*_), label *l*^*v*_*j*_^ is chosen, which satisfies *c*^*v*_*j*_^ = max(*c*^*v*_*k*_^ | (*l*^*v*_*k*_^, *c*^*v*_*k*_^) ∈ *B*(*v*_*j*_)), then node *v*_*j*_ sends label *l*^*v*_*j*_^ to node *v*_*i*_
2. When label *l*^*v*_*j*_^ reach node *v*_*i*_, it is assigned with label importance calculated by equation (7), then *B*(*v*_*i*_) = *B*(*v*_*i*_) ∪ (*l*^*v*_*j*_^, *LP*_*l*^*v*_*j*_^,*v*_*j*_→*v*_*i*__)
3. The label importance is added when the labels with the same id reach node *v*_*i*_

**Step 5 .**

Label acceptation. This step is used to accept useful labels and filter the labels with small belonging coefficients.

1. By normalizing the label importance of labels in *B*(*v*_*i*_), *B*(*v*_*i*_) = {(*l*_1_^*i*^, *c*_1_^*i*^), ⋯, (*l*_*j*_^*i*^, *c*_*j*_^*i*^), ⋯, (*l*_*H*_^*i*^, *c*_*H*_^*i*^)}, *c*_*j*_^*i*^ = *LP*_*l*_*j*_^*i*^_/∑_*k*=1_^*H*^*LP*_*l*_*k*_^*i*^_
2. For label (*l*_*j*_^*i*^, *c*_*j*_^*i*^) in *B*(*v*_*i*_), if *c*_*j*_^*i*^ < 1/*R*, then *B*(*v*_*i*_) = *B*(*v*_*i*_) − (*l*_*j*_^*i*^, *c*_*j*_^*i*^). The updated *B*(*v*_*i*_) of node *v*_*i*_ is gained by normalizing again, then the updating of labels of node *v*_*i*_ is finished. Here, *R* is the filtering threshold
3. If *r* = *N*_node_, then step 6 is executed, else the method sets *r* = *r* + 1, *S* = *S* − {*v*_*i*_} and returns to Step 2 to update other nodes.

**Step 6 .**

Termination judgement. The minimal number set *m*_*t*_ of nodes signed by each community identifier is computed. If *m*_*t*_ = *m*_*t*−1_ or LILPA reaches the maximum number of iterations, LILPA goes to Step 7 for postprocessing, else sets $S=V,{\vec{D}}_{v_{i}}=\vec{0},r=1,t=t+1$ and returns to Step 2 for the next iteration.

**Step 7 .**

Postprocessing. Nodes with label *l* are allocated to community *O*^*l*^. If nodes have multiple labels, then they are assigned to multiple communities.

We apply LILPA to herbal semantic network and discover herb community set *O* = {*O*^1^, ⋯, *O*^*i*^, ⋯, *O*^*k*^}, where *k* is the number of herb communities. In each community *O*^*i*^, herbs have the same or similar efficacy for treating multiple syndromes of a certain disease. Then, we can discover core herbs for treating the syndromes by choosing nodes with large degree in community *O*^*i*^.

## 4. The Proposed Model

In this paper, we aim to import herb knowledge implied in large-scale literature into core herb discovery. Thus, we propose CHDSC to analyse the semantics of herbs in literature based on semantic analysis module ESSP2VEC, calculate the semantic similarity among herbs to build herbal semantic network, and discover herb communities and core herbs in the network based on community detection module LILPA. CHDSC includes three stages: corpus construction, herb network establishment, and core herb discovery, whose process is shown in Figure 6.

Before applying CHDSC to discover core herbs for treating a certain disease, we should choose a target disease; here, we denote the target disease as *T*. After discussing with TCM experts, we select keywords in Chinese about the TCM treatment of disease *T* to search scientific literature in CNKI.

### 4.1. Corpus Construction

In this stage, corpus *C* about the TCM treatment of disease *T* is built by preprocessing the collected literature, which is used to train ESSP2VEC for analysing the semantics of herbs in literature.

**Step 8 .**

Word segmentation. Different from English sentences that use space as the natural interval among words, Chinese sentences are made up of continuous words. In order to analyse the semantics of Chinese words in literature, in this paper, Chinese sentences of the full text of literature are divided into Chinese words.

**Step 9 .**

Font conversion. Since traditional Chinese characters may exist in the literature, we convert them into simplified Chinese characters to make uniform the process.

**Step 10 .**

Redundant information removal. This step is to remove messy code, punctuations, and English abstract to obtain the pure corpus *C*, whose number of words is *N*_word_.

### 4.2. Herb Network Establishment

In this stage, herbal semantic network *G* is constructed by extracting the semantic word vectors of herbs and calculating their semantic similarity to reflect the relations between herbs and the target disease.

**Step 11 .**

Semantic analysis. Corpus *C* is input into ESSP2VEC to analyse the semantics of words in literature. Then, we obtain the semantic word vectors *U*.

**Step 12 .**

Name entity recognition. All Chinese words in the corpus including symptoms, syndromes, diseases, herbs, and other words are used to train word embedding because the semantics of herbs are contained in the contexts of words [38]. Then, the results contain the semantic word vectors of symptoms, syndromes, diseases, herbs, and other words. In this step, the semantic word vectors *U*_*X*_ of herbs is extracted from *U* by name entity recognition, where *X* represents the herbs existing in the collected literature. We construct a standard herbal name dictionary *D* according to the regulated herb name in *The Pharmacopoeia of the People's Republic of China* [52]. If herbs exist in the corpus and the standard herb thesaurus simultaneously, then we extract the herbs and their semantic word vectors.

**Step 13 .**

Semantic similarity calculation. Here, we adopt cosine similarity [53] to measure the semantic similarity among herbs, which is defined as

(12) $$\begin{array}{c} Q\left(w_{i},w_{j}\right)=\frac{u_{i}\cdot u_{j}}{\left|u_{i}\right|\left|u_{j}\right|}. \end{array}$$

If the semantic similarity among herbs is greater than the average value of all similarities among herbs, we consider that they own similar efficacy and can treat some syndromes of a disease.

**Step 14 .**

Herb network establishment. Herb semantic network is constructed by herbs and their semantic similarity. The herbs form nodes in the network, and if the similarity of two herbs is greater than the average value of all similarities among herbs, then an edge is formed between the two herbal nodes.

### 4.3. Core Herb Discovery

In this stage, core herb set *D*^core^ = {*D*_1_^core^, ⋯, *D*_*i*_^core^, ⋯, *D*_*k*_^core^} is discovered in herb community *O* = {*O*^1^, ⋯, *O*^*i*^, ⋯, *O*^*k*^}.

**Step 15 .**

Herb community discovery. Herbs in herb communities own the same or similar efficacy to treat multiple syndromes of a disease. Herb communities are revealed by LILPA.

**Step 16 .**

Core herb discovery. In each community, nodes are important if they have a large degree. We choose eight herbs with top-8 degree in each community as core herbs.

### 4.4. Complexity Analysis

The complexity of CHDSC is mainly in the two artificial intelligence modules. Here, we briefly analyse the time complexity of ESSP2VEC and LILPA.

#### 4.4.1. The Time Complexity of ESSP2VEC

The contextual words are predicted based on each word taking time *O*(*cN*_word_). We adopt an optimal strategy, negative sampling [45], which considers the target word and its contextual words as positive sample pairs and takes the target word and random words as negative sample pairs, whose number is *N*_neg_. Then, the problem of predicting contextual words can be replaced as a set of independent binary classification tasks so as to independently predict the presence (or absence) of contextual words [39] [40]. Then, equation (3) can be rewritten as

(13) $$\begin{array}{c} p\left(w_{c}\;|\;w_{t}\right)=\frac{e^{s\left(w_{t},w_{c}\right)}}{\sum_{j=1}^{c+N_{\text{neg}}}e^{s\left(w_{t},w_{j}\right)}}. \end{array}$$

Thus, the complexity of predicting the contextual words of a word can be reduced to *O*(*c*(*c* + *N*_neg_)). Then, predicting the contextual words of all words costs time *O*(*c*(*c* + *N*_neg_)*N*_word_). For ESSP2VEC, we represent each word as its stroke *n*-gram with structure and pinyin features and predict the contextual words based on the ensemble features of the target word, then the total complexity is *O* ((*L*_max_(*L*_max_ + 1)/2) *c*(*c* + *N*_neg_)*N*_word_), where *L*_max_ is the maximum length of stroke *n*-gram. In general, *c*, *N*_neg_, *L*_max_ ≪ *N*_word_, then the total complexity is near *O*(*h*_1_*N*_word_), where *h*_1_ is a constant.

#### 4.4.2. The Time Complexity of LILPA

The time complexity of LILPA is estimated as follows.

1. *Initialization*: the shortest distances among nodes are calculated with time *O*(*N*_node_log*N*_node_). The Quicksort algorithm is adopted for sorting nodes by node importance with time *O*(*N*_node_log*N*_node_). Thus, initialization costs time *O*(*N*_node_log*N*_node_)
2. *Node choice*: choosing a node to update its label costs constant time
3. *Node movement*: calculating the attractive and repulsive forces between node *v*_*i*_ and its neighbours and the displacement of node *v*_*i*_ takes time *O*(∣*N*(*v*_*i*_)∣)
4. *Label launch*: the neighbours of node *v*_*i*_ cost the worst time *O*(∣*N*(*v*_*i*_) | *n*_1_log*n*_1_) to send their labels, where *n*_1_ is the maximum number of labels of the neighbours of node *v*_*i*_. In general, *n*_1_ ≪ *N*_node_, then label launch needs constant time
5. *Label acceptation*: accepting the labels of node *v*_*i*_ takes *O*(*n*_2_), where *n*_2_ is the number of labels reaching node *v*_*i*_. In general, *n*_2_ ≪ *N*_node_, then label acceptation takes constant time
6. *Termination judgement and postprocessing*: the same as COPRA [54], the former costs time *O*(*βN*_node_) and the latter needs time *O*((*β*^3^ + 1)*N*_node_ + *β*(*N*_node_ + *M*_edge_))

For the label update process of node *v*_*i*_, Steps 2–5 need constant time. Thus, updating the labels of *N*_node_ nodes in one iteration needs time *O*(*N*_node_). Thus, the time complexity of LILPA is *O*(*N*_node_log*N*_node_ + (*β*^3^ + 2*β* + *t* + 1)*N*_node_ + *βM*_edge_). In general, *β*, *t* ≪ *N*_node_, *M*_edge_, then the total complexity is near *O*(*N*_node_log*N*_node_ + *h*_2_*N*_node_ + *h*_3_*M*_edge_), where *h*_2_ and *h*_3_ are constants.

## 5. Experiment Setup

In this section, we first introduce datasets, evaluation criteria, and comparison algorithms, which are used to evaluate the performance of artificial intelligence modules. Then, we take a case study by choosing CGN as the target disease and apply CHDSC to discover the core herbs for treating multiple syndromes of CGN in TCM.

### 5.1. Data Description

For evaluating the effectiveness of the semantic analysis module (i.e., word embedding algorithm ESSP2VEC), we employ a universal data SogouCA shown in Table 2, which contains 300 million words after preprocessing by the same operation of corpus construction to train ESSP2VEC to obtain word semantic vectors. Then, we use datasets (1) WA-1124, (2) WS-240, and (3) WS-296 to evaluate the proposed module on word analogy and word similarity tasks, respectively, as described in Section 5.2. For estimating the performance of community detection module (i.e., label propagation algorithm LILPA), we use eight real-world networks shown in Table 3. Each algorithm independently runs 50 times.

### 5.2. Evaluation Criteria

In order to evaluate the quality of semantic word vectors obtained by word embedding algorithms, we test them on word analogy and word similarity tasks.

- Word analogy task is used to measure the model ability of exploring the semantic relations among words [42] [45]. Given three words *w*_1_, *w*_2_, and *w*_3_, the word embedding models judge word *w*_4_ that correctly answers the question “*w*_1_ to *w*_2_ is *w*_3_ to what?” For example, there is a question “*Beijing* is to *China* as *Berlin* is to what?” such that the cosine similarity between vectors (*v*_*w*_2__ − *v*_*w*_1__ + *v*_*w*_3__) and *v*_*w*_4__ is maximized. By correctly answering this question, such as *Germany*, the models are considered that they can capture semantic relationships among words. We adopt the test data WA-1124 with 1124 instances for evaluating Chinese word semantic vectors [42]
- Word similarity task is designed to evaluate the model ability of capturing semantic relatedness and closeness among words [39] [40]. Word similarity is measured by the cosine similarity between the corresponding word vectors, then we calculate the Spearman correlation coefficient between the word similarity and the human similarity scores to estimate the quality of word vectors. We adopt two datasets WS-240 and WS-296 for evaluation [39]

In order to measure the quality of detected communities in networks, we use two criteria Normalized Mutual Information (NMI) and Overlap Modularity (OM). If the true communities of real-world networks are known, the two criteria are both adopted; otherwise, only OM is adopted.

- NMI is used to compute the difference between the communities detected by algorithms and true community structures and varies between 0 and 1 [62]. The larger the value, the smaller the difference
- OM reflects the quality of divisions assessed by the relative density of edges within communities and between communities [63], which varies between 0 and 1. The larger the value, the better the quality

### 5.3. Comparison Algorithms

To evaluate the effectiveness of ESSP2VEC, we compare it with seven word embedding algorithms, including (1) three general word embedding algorithms CBOW [45], Skip-Gram [45], and GloVe [64], which can be used for any languages, and (2) four Chinese word embedding algorithms CWE [42], JWE [44], GWE [65], and CW2VEC [39], which are designed for the Chinese language and consider the radical, component, character, and stroke *n*-gram features, respectively. For baselines, we set the size of the contextual window equalling to ESSP2VEC.

To show that LILPA can find better communities, we compare it with seven label propagation-based community detection algorithms COPRA [54], SLPA [66], DLPA^+^ [67], WLPA [68], LPA_NI [69], NGLPA [70], and LPANNI [49]. In this paper, we use the given parameters for baselines if real-world networks are used in the original articles. Otherwise, we utilize the ways proposed in the original articles to gain the best solution.

### 5.4. Case Study

In order to further validate the effectiveness of core herb discovery model CHDSC, we choose CGN as the target disease to conduct a case study. After discussing with TCM experts, we select keyword pairs in Chinese (1) “chronic glomerulonephritis” and “Chinese medicine” and (2) “chronic glomerulonephritis” and “Chinese native medicine,” to search the scientific literature in CNKI. Then, we apply CHDSC to analyse the collected literature to discover the core herbs for treating different syndromes of CGN.

## 6. Results and Discussion

The results for word analogy and word similarity tasks are shown in Table 4. The average values of NMI and OM for real-world networks are shown in Tables 5 and 6, respectively. We mark the optimal values in italics. The number in brackets is the rank of methods for each task or network, and the average rank of each algorithm is shown in the last column. Finally, we choose CGN as the target disease to conduct a case study.

### 6.1. Results of Word Embedding Algorithm

As shown in Table 4, we can find that ESSP2VEC obtains the best result in all tasks. For word analogy task, CBOW and Glove achieve about 20% accuracy, CWE and GWE obtain over 40% accuracy, Skip-Gram and JWE gain over 50% accuracy, and the accuracy of CW2VEC and ESSP2VEC is over 60%. In general, the proposed algorithm ESSP2VEC outperforms the best baseline CW2VEC. For word similarity task in terms of WS-240, CBOW and Glove gain over 40% accuracy and other algorithms achieve over 50% accuracy. ESSP2VEC outstrips the best baseline Skip-Gram. For word similarity in terms of WS-296, the accuracy of CBOW and Glove is under 60%; on the contrary, other algorithms obtain over 60% accuracy. ESSP2VEC outperforms the best baseline CW2VEC. Thanks to the ideas of using the target word to predict its contexts and the effectiveness of integrating the stroke, structure, and pinyin features of Chinese characters, ESSP2VEC obtains the best average rank on word analogy and word similarity tasks. Comparing with state-of-the-art word embedding algorithms, we can consider that the proposed algorithm ESSP2VEC can obtain good accuracy and analyse the semantics of herbs in the literature.

### 6.2. Results of Label Propagation-Based Algorithm

As shown in Table 5, we can find that LILPA obtains the best NMI for the Karate, Dolphins, and Football networks and achieves the best average rank, which illustrates that LILPA can discover communities close to the true ones. In particular, LILPA outperforms the best baseline LPANNI over 20.73% for the Karate network and outstrips the best baseline NGLPA over 10.17% for the Dolphins network. Although LILPA obtains poor NMI than some algorithms for the Netscience network, the difference with the optimal value is small. As shown in Table 6, LILPA gains the first rank in five networks and the second rank in two networks, then it achieves the best average rank. LILPA gets poor OM in the Dolphins network, while it obtains the best NMI in this network. With the increase of network scale, LILPA keeps good performance. LILPA can find better communities in different scale networks than other baselines. In general, according to the average rank, LILPA outperforms baselines in terms of NMI and OM, which is profited by node importance, node attraction, and label importance. Compared with state-of-the-art label propagation-based algorithms, we can infer that LILPA can discover good communities and can detect high-quality herb communities in the herbal semantic network.

### 6.3. Results of the Application of CHDSC on CGN

In this section, we choose CGN as the target disease *T* for the reason mentioned in Section 1. According to the above experiments, we can consider that CHDSC with ESSP2VEC and LILPA can discover core herbs accurately. Then, we apply CHDSC to discover core herbs for CGN treatment in TCM. After searching the literature in CNKI, we collect 449 samples of literature by keywords “chronic glomerulonephritis” and “Chinese medicine” and 677 samples of literature by keywords “chronic glomerulonephritis” and “Chinese native medicine.”

After corpus construction, we obtain CGN corpus containing 1126 samples of literature with 0.8 million words. All articles are related to the TCM treatment of CGN, so we expect semantic analysis can obtain high-quality semantic word vectors of herbs, since a pure in-domain corpus yields better performance than a mixed-domain corpus [71].

After herb network establishment, we obtain the semantic word vectors of 274 herbs and build a herbal semantic network with 274 nodes and 1293 edges. Some nodes have no edges with others because these herbs may have small similarity with other herbs. In order to understand the semantic word vectors intuitively, we choose two herbs *dwarf lilyturf tuber* (Mai Dong) and *combined spicebush root* (Wu Yao), discover the herbs owing large semantic similarity with one of them, and visualize these herbs in a two-dimensional surface. As shown in Figure 7, *dwarf lilyturf tuber* (Mai Dong) and some herbs are clustered together (denoted as *O*^1^ with red color), and *combined spicebush root* (Wu Yao) and some herbs are also gathered together (denoted as *O*^2^ with green color). Meanwhile, we can observe that groups *O*^1^ and *O*^2^ have obvious interval, then we can infer that the semantic word vectors of *dwarf lilyturf tuber* and *combined spicebush root* can reflect their characteristics to find similar herbs. CHDSC can capture the semantics of herbs in the literature to a certain extent and generate effective semantic word vectors.

After core herb discovery, CHDSC discovers three large herb communities in herbal semantic network as shown in Figure 8. The herbs in the same community own similar efficacy and can treat multiple syndromes of CGN. According to the analysis of TCM experts, the herbs in the blue community have the efficacies of nourishing the liver and kidney and nourishing yin and blood, which can be mainly used for treating the syndrome of deficiency of both qi and yin and the syndrome of yin deficiency of the liver and kidney. The herbs in the purple community have the efficacies of removing dampness and diuresis, clearing heat and removing toxicity and dispelling wind evil and are often used for treating the syndrome of yang deficiency of the spleen and kidney. Meanwhile, they can be used to treat the syndromes of dampness-heat and fluid-dampness. The herbs in the green community have the efficacies of activating qi and eliminating dampness, clearing heat and removing toxicity, and resolving masses, which are used to treat the syndrome of liver depression and qi stagnation. According to the pathogenesis of CGN in TCM (intermingled deficiency and excess) and the TCM treatment points for CGN (supple deficiency and expel excess and strengthening vital qi to eliminate pathogenic factor) [36, 37], we find that the herbs in the blue community are mainly used for supplying deficiency and the herbs in the purple and green communities are mainly used for expelling excess. Thus, the herbs in the blue community are necessary for treating CGN in TCM, and the ones in the purple and green communities are used to treat the secondary symptoms. CHDSC discovers herb communities where herbs can treat most primary syndromes of CGN; however, herbs in herb communities do not cover all syndromes of CGN, which may be because some syndromes are less recorded in the literature and the scale of the literature is limited.

The herbs represented by the nodes with the top-8 degree in each community are regarded as core herbs for treating multiple syndromes of CGN as shown in Figure 9 (their Chinese pinyin and English name are shown in Tables 7–9). According to the analysis of TCM experts, for the herbs with the top-8 degree, the herbs in red circles are the core herbs identified correctly for treating the CGN syndromes represented by corresponding herb communities and the herbs in yellow circles are complementary herbs (the core herbs identified correctly are indicated in italics in Tables 7–9). It is seen that CHDSC can discover core herbs for treating most syndromes of CGN with high accuracy from large-scale literature, which can give references for the clinical application of herbs. Thus, we can consider that CHDSC can automatically discover core herbs for treating a disease from large-scale literature. The herbs in red circles are core herbs and can be used to treat main symptoms of CGN; the herbs in yellow circles are used to play support efficacy according to the symptoms of patients because patients may suffer from other diseases and need to be treated at the same time.

In order to further explore the herbal semantic network, we analyse its community size, degree, and closeness centrality distributions to mine the rules of CGN core herbs.

- Community size distribution can reflect the community number of networks and the number of nodes in each community
- Degree distribution can measure the number of nodes with different degrees
- Closeness centrality distribution can reflect the number of nodes with different closeness. The closeness centrality of a node is a measure of centrality in a network. The more central a node is, the closer it is to other nodes

The results are shown in Figure 10, and the degree and closeness centrality values of core herb nodes are shown in Tables 7–9. As shown in Figure 10(a), there are three large communities, in which each community owns more than 25 nodes. Other communities are small and only have few nodes because the literature records complex symptoms and syndromes, and these herbs in small communities are used to treat other symptoms of patients. Thus, core herbs are discovered from the three communities for treating the main symptoms and syndromes of CGN in TCM. As shown in Figures 10(b) and 10(c) and Tables 7–9, the degree and closeness centrality of core herb nodes concentrate on the range of [15, 40] and [0.25, 0.45], respectively. It suggests that core herbs are represented by the important and central nodes in the herb network. Thus, if we construct a new herb network from new literature, then we can prejudge the core herbs for treating CGN according to their degree and closeness centrality, which can reduce cost and increase accuracy. For other diseases, we also can utilize the above rules to prejudge core herbs according to their degree and closeness centrality. So, these circled states can reflect the distribution rules of core herbs and are important for doctors and researchers to explore core herbs for CGN and other diseases.

## 7. Conclusions

In this paper, we study the problem of core herb discovery in TCM and propose an artificial intelligence model CHDSC to discover core herbs for treating a certain disease from large-scale literature based on semantic analysis and community detection, in which word embedding algorithm ESSP2VEC is designed to analyse the semantics of herbs in the literature, and label propagation-based algorithm LILPA is used to discover herb communities and core herbs. In the case study, CHDSC discovers three large herb communities where herbs can treat most syndromes of CGN and identifies core herbs for treating these syndromes with high accuracy. CHDSC can discover effective core herbs, which is helpful for the clinical application of herbs and formulae. In addition, the proposed model is introduced to discover core herbs for treating CGN as an example; it also can be applied to other diseases.

We also find that some syndromes cannot be covered by discovered core herbs and some core herbs with low degree (e.g., *asiatic cornelian cherry fruit* (Shan Zhu Yu) in blue community) are not discovered. These syndromes may be less recorded in the literature, and the collected literature may not contain the usage of these core herbs in most cases. Improving the semantic analysis and community detection modules is an important area of future research. For example, importing the “Sovereign-Minister-Assistant-Courier” combination rule in LILPA can combine TCM domain knowledge with community detection to guide label propagation and form a supervised way. The source and scale of literature have the influence on results, so enlarging the scale of the corpus and selecting authoritative literature can enhance the accuracy. In addition, for the Chinese word embedding algorithm ESSP2VEC, we can consider the syntax and Part of Speech (POS) [72] as features and predict the contextual words based on soft tree [73] to learn the semantics of Chinese words, which will also be the subject of future research.

## Figures and Tables

**Figure 1:** The framework of CHDSC. CHDSC consists of two modules, semantic analysis and community detection, in which the former is a Chinese word embedding algorithm ESSP2VEC to analyse the semantics of herbs and the latter is a label propagation-based algorithm LILPA to detect herb communities and core herbs. As a case study, we take CGN as an example and discover core herbs to treat different syndromes of CGN.

**Figure 2:** Example of semantic word vectors.

**Figure 3:** The architecture of ESSP2VEC. First, we decompose a Chinese word to characters and extract their stroke, structure, and pinyin features in the feature extraction layer. Second, the three features are encoded in the feature encoding layer. Third, we generate stroke *n*-gram and integrate stroke *n*-gram, structure, and pinyin features in the ensemble feature layer. Finally, the contextual words are predicted based on the ensemble features of the target word to learn the semantics of the target word.

**Figure 4:** Example of label propagation for community detection.

**Figure 5:** The process of LILPA. LILPA first initializes each node with a unique label, chooses nodes to update according to node importance, and moves nodes in the layout area according to node attraction. Then, the neighbour nodes of the updating node launch labels, and the updating node accepts labels according to label importance. The above steps except initialization are iteratively executed until all nodes are updated once. If LILPA reaches termination condition, then it goes to postprocessing, else, it returns to the step of node choice for the next iteration.

**Figure 6:** The process of CHDSC.

**Figure 7:** Example of semantic word vectors of herbs.

**Figure 8:** Results of herb communities.

**Figure 9:** Results of core herbs in each community. Herbs in red circles are the core herbs identified correctly for treating multiple syndromes of CGN. Herbs in yellow circles are complementary herbs.

**Figure 10:** Results of network distributions.

**Algorithm 1:** CHDSC.

**Table 1:** Corresponding concepts.

Core herb discovery	LILPA
Herb	Node
The relations among herbs	Edge
Efficacy	Label
Herb group for treating multiple syndromes	Community
Core herbs for treating multiple syndromes	Nodes with a top-*k* degree in each community

**Table 2:** Description of training and evaluation dataset.

Function	Dataset	Reference	Task	Scale
Training	SogouCA	[40]	—	300 million words
Evaluation	WA-1124	[42]	Word analogy	1124 instances
	WS-240	[39]	Word similarity	240 instances
	WS-296	[39]	Word similarity	296 instances

**Table 3:** Description of real-world networks.

Network	*N*_node_	*M*_edge_	*N*_com_	<*k*>	Dia	Reference
Karate	34	78	2	4.588	5	[55]
Dolphins	62	159	2	5.129	8	[56]
Football	115	615	12	10.661	4	[57]
Netscience	1589	2742	16	3.451	17	[58]
Power	4941	6594	–	2.669	46	[59]
PGP	10680	24316	–	4.554	24	[60]
Cond2003	31163	120029	–	7.703	16	[61]
Cond2005	40421	175693	–	8.693	18	[61]

*N*_com_: the number of communities; <*k*>: the average degree of networks; dia: the diameter of networks.

**Table 4:** Results of word analogy and word similarity tasks.

Algorithm	Word analogy (%)	Word similarity (%)		Average rank
	WA-1124	WS-240	WS-296	
CBOW	22.77 (7)	46.40 (8)	56.26 (7)	7.33
Skip-Gram	58.45 (3)	55.36 (2)	60.76 (4)	3.00
Glove	19.39 (8)	48.36 (7)	47.02 (8)	7.67
CWE	47.69 (6)	51.67 (5)	61.17 (3)	4.67
JWE	57.65 (4)	51.00 (6)	60.22 (6)	5.33
GWE	48.84 (5)	53.45 (4)	60.63 (5)	4.67
CW2VEC	63.17 (2)	54.85 (3)	61.41 (2)	2.33
ESSP2VEC	*64.85 (1)*	*55.38 (1)*	*61.71 (1)*	*1.00*

**Table 5:** Average value of NMI.

Algorithm	Karate	Dolphins	Football	Netscience	Average rank
COPRA	0.3596 (8)	0.5976 (6)	0.8836 (7)	0.3566 (5)	6.5000
SLPA	0.6915 (3)	0.6678 (3)	0.8862 (6)	0.3651 (2)	3.5000
DLPA^+^	0.5489 (5)	0.4753 (8)	0.9044 (2)	*0.3858 (1)*	4.0000
WLPA	0.5016 (6)	0.6599 (4)	0.9013 (3)	0.3350 (8)	5.2500
LPA_NI	0.6598 (4)	0.6436 (5)	0.8823 (8)	0.3636 (3)	5.0000
NGLPA	0.4408 (7)	0.7108 (2)	0.8887 (5)	0.3471 (7)	5.2500
LPANNI	0.7782 (2)	0.5809 (7)	0.8997 (4)	0.3627 (4)	4.2500
LILPA	*0.9855 (1)*	*0.8125 (1)*	*0.9079 (1)*	0.3526 (6)	*2.2500*

**Table 6:** Average value of OM.

Algorithm	Karate	Dolphins	Football	Netscience	Power	PGP	Cond2003	Cond2005	Average rank
COPRA	0.2348 (8)	0.3741 (7)	0.5972 (6)	0.8784 (7)	0.1696 (8)	0.5117 (8)	0.6306 (5)	0.4256 (8)	7.1250
SLPA	0.3742 (5)	0.4757 (5)	0.6016 (3)	0.9043 (6)	0.6225 (6)	0.7641 (4)	0.6341 (2)	0.6019 (5)	4.5000
DLPA^+^	0.4210 (2)	0.5166 (3)	0.5960 (7)	0.8456 (8)	0.5993 (7)	0.6761 (6)	0.4764 (8)	0.4371 (7)	6.0000
WLPA	0.3682 (6)	0.3695 (8)	0.5981 (5)	0.9279 (2)	0.7731 (2)	0.6231 (7)	0.5959 (6)	0.6117 (3)	4.8750
LPA_NI	0.4136 (4)	0.5055 (4)	0.5985 (4)	0.9140 (4)	0.7473 (4)	0.7861 (3)	0.6313 (3)	0.6111 (4)	3.7500
NGLPA	0.3314 (7)	0.5189 (2)	0.5848 (8)	0.9209 (3)	0.7631 (3)	*0.8092 (1)*	0.5907 (7)	0.4431 (6)	4.6250
LPANNI	0.4147 (3)	*0.5423 (1)*	*0.6090 (1)*	0.9070 (5)	0.6608 (5)	0.7575 (5)	0.6312 (4)	0.6175 (2)	3.6250
LILPA	*0.4213 (1)*	0.4003 (6)	0.6061 (2)	*0.9319 (1)*	*0.7817 (1)*	0.8001 (2)	*0.6852 (1)*	*0.6223 (1)*	*1.8750*

**Table 7:** Top-8 herbs in blue community.

Herb (Chinese pinyin)	Herb (English name)	Degree	Closeness centrality
*Sha Shen*	*Coastal glehnia root*	*26*	*0.35*
Bu Gu Zhi	Malaytea scurfpea fruit	25	0.33
Sang Ji Sheng	Chinese taxillus herb	23	0.35
*Mai Dong*	*Dwarf lilyturf tuber*	*22*	*0.34*
*Nv Zhen Zi*	*Glossy privet fruit*	*20*	*0.30*
*Lu Jiao Jiao*	*Deerhorn glue*	*17*	*0.31*
*Shu Di Huang*	*Prepared rehmannia root*	*15*	*0.28*
*Bai Shao*	*Debark peony root*	*15*	*0.34*

**Table 8:** Top-8 herbs in purple community.

Herb (Chinese pinyin)	Herb (English name)	Degree	Closeness centrality
*Tong Cao*	*Ricepaperplant pith*	*39*	*0.40*
*Xuan Shen*	*Figwort root*	*35*	*0.39*
Sheng Jiang	Fresh ginger	34	0.38
Ren Dong Teng	Honeysuckle stem	33	0.41
*Chen Pi*	*Dried tangerine peel*	*32*	*0.39*
*Yu Jin*	*Turmeric root tuber*	*32*	*0.40*
*Mu Dan Pi*	*Tree peony root bark*	*29*	*0.41*
*Jie Geng*	*Platycodon root*	*28*	*0.37*

**Table 9:** Top-8 herbs in green community.

Herb (Chinese pinyin)	Herb (English name)	Degree	Closeness centrality
*Wu Yao*	*Combined spicebush root*	*48*	*0.42*
Sheng Ma	Largetrifoliolious bugbane rhizome	36	0.38
*Bian Xu*	*Common knotgrass herb*	*35*	*0.32*
Mo Yao	Myrrh	35	0.34
*Zhen Zhu Mu*	*Nacre*	*34*	*0.34*
*Lu Gen*	*Reed rhizome*	*33*	*0.38*
*Lu Xian Cao*	*Pyrola herb*	*23*	*0.31*
*Qing Pi*	*Immature tangerine peel*	*23*	*0.38*

## Data Availability

The text data used to support the findings of this study have been deposited in https://github.com/yunzhangwww/TCM-literature-corpus
